The article "Potential Factors for Psychological Symptoms at Three Months in Patients with Young Ischemic Stroke" was retracted in 2024. Reasons: signs of a paper mill; suspected computer-generated content; unreliable results or conclusions; concerns about the data.

# Potential Factors for Psychological Symptoms at Three Months in Patients with Young Ischemic Stroke

**DOI:** 10.1155/2021/5545078

**Published:** 2021-02-09

**Authors:** Dongjuan Xu, Xi Chu, Kun Wang, Lianyan Wei, Yunyun Xu, Xiaomin Huang, Jinna Li, Lina Xu, Lu Yin, Hong Liu, Xiaolei Liu, Haixia Leng, Qing Xue, Mao Peng, Longbin Jia, Hongxing Wang

**Affiliations:** ^1^Department of Neurology, Dongyang People's Hospital, Wenzhou Medical University, Zhejiang, China 322100; ^2^Health Management Department, Xuanwu Hospital, Capital Medical University, Beijing, China 100053; ^3^Department of Neurology, Beijing Puren Hospital, Beijing, China 100062; ^4^Department of Neurology, Xuanwu Hospital, Capital Medical University, Beijing, China 100053; ^5^Department of Neurology, Ningcheng Center Hospital, Inner Mongolia, China 024200; ^6^Department of Neurology, Jincheng People's Hospital, Shanxi, China 048026; ^7^Medical Research & Biometrics Centre, National Centre for Cardiovascular Diseases, Fuwai Hospital, Peking Union Medical College & Chinese Academy of Medical Sciences, Beijing, China Beijing, China 102300; ^8^Department of Neurology, Heping Hospital Affiliated to Changzhi Medical College, Shanxi, China 046000; ^9^Department of Neurology, The First Affiliated Hospital of Kunming Medical University, Yunnan, China 650032; ^10^Beijing Psychosomatic Disease Consultation Center, Xuanwu Hospital, Capital Medical University, Beijing, China 100053; ^11^Institute of Sleep and Consciousness Disorders, Beijing Institute for Brain Disorders, Capital Medical University, Beijing, China 100053

## Abstract

**Objective:**

Psychological status plays a vital role in the recovery in young ischemic stroke patients. However, few reports on the psychological symptoms in Chinese young ischemic stroke patients have been published. In the present study, we aimed to outline the psychological status of young ischemic stroke patients and its risk factors at three months after their stroke.

**Methods:**

364 patients with young ischemic stroke and 384 age-matched healthy controls were consecutively recruited from our study hospitals of the mainland of China between June 2018 and November 2020. Social demographic and clinical data were collected from all enrolled participants in the acute stage of their stroke, and their psychological variables were assessed via the Symptom Checklist 90 Revised (SCL-90-R) at three-month timepoint after their stroke. Multivariable logistic regression analyses were run to identify the independent factors for psychological variables in patients.

**Results:**

Compared with healthy controls, patients with young ischemic stroke had significantly higher total score of SCL-90-R and all subscale total scores (*p* < 0.01 or 0.05). 22.3% (81/364 cases) in young ischemic stroke patients had psychological abnormalities. Compared with young ischemic stroke patients without psychological symptoms (*n* = 283), patients with psychological symptoms (*n* = 81) had higher rate of married status (*p* = 0.03), rate of hypertension (*p* = 0.01), infarct size (*p* = 0.01), and the family dysfunction (*p* < 0.01). Multivariate logistic regression analyses revealed that the family dysfunction (odds ratio [OR], 2.50, 95% confidence interval [CI]: 1.71 to 3.54, *p* < 0.01), having hypertension (OR, 3.27, 95% CI: 1.92 to 4.27, *p* = 0.02), and ≥20mm^3^ infarct size (OR, 2.39, 95% CI: 1.53 to 3.45, *p* < 0.01) were independent factors for having psychological abnormalities in patients with young ischemic stroke at three months after their stroke. Single (OR, 1.23, 95% CI: 1.03 to 1.54, *p* = 0.01), poor family function (OR, 1.21, 95% CI: 1.05 to 1.45, *p* = 0.03), and ≥20mm^3^ infarct size (OR, 1.74, 95% CI: 1.14 to 3.13, *p* = 0.02) were independent factors for having depression in patents with psychological symptoms. The family dysfunction (OR, 2.32, 95% CI: 1.51 to 2.80, *p* < 0.01) and hypertension (OR, 2.41, 95% CI: 1.54 to 3.46, *p* = 0.03) were independent factors for emerging somatization and anxiety in patients with psychological symptoms, respectively.

**Conclusions:**

At three months after their stroke, young ischemic stroke patients had psychological problems and risk factors for developing them.

## 1. Introduction

Stroke is one leading cause of death in adults worldwide [1, 2] and is one of the main causes of death and a significant contributor to disability in adults in China, characterized by high rates of morbidity, fatality, and disability, bringing a severe economic burden [3–5]. Among the stroke population, the incidence of stroke in older adults decreases while the incidence of young adult stroke is increasing, around 1 in 10 about a young adult [1]. Youth adult stroke often occurs in adults aged 18 to 60 years, especially 18 to 45 years [6]. Moreover, there is a trend that stroke occurs in individuals at a younger age [6, 7]. Most importantly, stroke in young adults has a considerable socioeconomic influence associated with high health-care costs and tremendous loss of labor productivity [4, 6, 8, 9]. Therefore, any potential characteristics of the young adults' stroke still need to be further emphasized [10].

The negative emotion is one of the most symptoms emerging in patients with stroke [10, 11]. Unfortunately, the current optimal management of young adult patients with stroke, unlike treatment for older adults, is unknown [1, 12]. The available recovery strategy for young stroke patients does not provide psychological intervention [10]. The related risk factors on young adult patients have been summarized in the recent review [1], as there is no report on the psychological symptoms and its risk factors in young ischemic stroke patients.

The recovery for young ischemic stroke patients relies on not only physical rehabilitation but also psychological situation [1, 10, 13, 14]. Recent studies have shown that the poststroke psychological status plays a role in the recovery of young ischemic stroke patients in the clinical practice setting [10, 15], while family support and social support are important factors associated with psychological status for persons who can find assistance from outside when they need help [16–18]. These aforementioned studies suggest that the poststroke psychological level is necessarily explored in young ischemic stroke patients for their recovery. Here, we conducted a prospective study to investigate the psychological status and its risk factors in these populations.

## 2. Methods

### 2.1. Clinic Setting

All 364 patients and 384 age-matched healthy controls were consecutively recruited from our study hospitals and their health management departments, including 5 comprehensive hospitals of the mainland of China between June 2018 and November 2020. The study protocols were approved by the Local Ethics Committees of Xuanwu Hospital, Capital Medical University (LYS2018008) and Dongyang People's Hospital, Wenzhou Medical University (2017-KY-036 and 2018-YX-051). All subjects provided written informed consent. This research was conducted by the Helsinki Declaration.

### 2.2. Participants

Patients were consecutively enrolled the study if they met the following criteria: (a) aged 18 to 45 years, (b) satisfied the stroke diagnostic criteria formulated by the Chinese cerebrovascular disease classification and were confirmed by magnetic resonance imaging or computed tomography scan [19], (c) could answer questionnaires independently, and (d) knew his/her illness. The exclusion criteria were (a) presence of the other nonvascular causes (such as primary brain tumor, brain metastases, subdural hematoma, postictal paralysis, and brain trauma) related to brain dysfunction; (b) a previous history of depression, psychosis, and dementia; (c) could not understand and complete the examination; and (d) refused to provide written consent.

### 2.3. Measures

At the baseline (i.e., in the acute stage of stroke), the following basic data were collected. Social-demographic and clinical data were collected from all enrolled participants in the acute stage of their stroke, including age, sex, living area (i.e., urban and rural), education status (i.e., junior high school and lower, senior high school and higher), marital status (i.e., married, unmarried, divorced, and widowed), having medical insurance (yes or no), monthly income (>6,000 Yuan, ≤6,000 Yuan), smoke and drink dependence (yes or no), hypertension (yes or no), diabetes (yes or no), atrial fibrillation (yes or no), the National Institute of Health Stroke Scale (NIHSS) [20], the modified Rankin Scale (mRS) [21], the Barthel Index (BI), infarct location (i.e., cortex, white matter lesions, basal ganglia + thalamus, brain stem, and cerebellum) [22, 23], and infarct size (≥20 vs. <20 mm^3^) calculated in three days after stroke onset by manually delineating the hypodense infarcted area(s) on hyperintense area(s) on axial diffusion weighted imaging slices on magnetic resonance imaging (MRI) [24, 25].

At three-month time after their stoke, all participants' psychological state was evaluated. In details, the psychological status, family function, and social support were assessed via the Symptom Checklist 90 Revised (SCL-90-R), the family function assessment scale (FFAS), and the social support rating scale (SSRS) at three months after stroke, respectively. After obtaining written informed consent, as explained by our study alliance doctors, all participants were administered via the questionnaires for their clinical assessment. The qualified raters were trained to give information about the questionnaire to the participants, who were permitted to complete the questionnaire by themselves without time restriction and in a state where patients were willing to cooperate.

The SCL-90-R is a 5-point scale, 90-item self-report tool that measures the degree of symptoms on different dimensions such as somatization, obsessive-compulsive, depression, anxiety, phobic anxiety, hostility, interpersonal sensitivity, paranoid ideation, and psychoticism [26]. It is widely used to screen psychological symptoms, and the Chinese version of the SCL-90-R is reported [27] with favorable validity and reliability [28]. Higher scores indicate more significant psychological symptoms. For Chinese, the total score of SCL-90-R is over 160, which is regarded as the criteria of an individual who has abnormal psychological status [29]. The results on SCL-90-R of the study were compared with the previously reported standard models of 1986 [30] and 2006 [31].

FFAS is a 3-point scale (0-not at all, 1-sometimes, 2-often), 5 items self-report instrument to evaluate family functioning via five dimensions, including adaption, cooperation, growth, affection, and intimacy. The total score of FFAS is 10 points, and the higher total score indicates better family function. The criteria for a good family function, moderate impairment in family function, and severe impairment in family function are 7-10 points, 4-6 points, and 0-3 points of the FFAS total score, respectively [16].

SSRS is a 10-item self-reported tool that evaluates the degree of an individual's social support over the past year. The tool comprises three subscales: subjective support, objective support, and utilization of support [17]. Subjective support means perceived social support that individual feel supported, cared, and helped by his/her family members, friends, and colleagues (e.g., how many close friends do you have? (1) None, (2) 1-2, (3) 3-5, and (4) 6). Objective support refers to visible, practical, and direct support (e.g., the recourses where you got financial and reliable support when you needed help?). The employment of support means the level of social support applied (how do you get help when in need? (1) I am self-dependent. (2) I seldom ask for help from others. (3) I sometimes ask for help from others. (4) I often ask for help from my relatives and friends.). The SSRS total score ranges from 12 to 66 points, and higher scores on this tool indicate a higher degree of social support. The SSRS has been shown to have good reliability and validity, with Cronbach's *α* ranging from 0.825 to 0.896 [18]. The results of SSRS are classified into three different levels in our study. It is generally considered <20 points that indicate that the individual has obtained less social support, 20-30 points suggest that the individual has accepted general social support, and >30 points indicate that the individual has received satisfactory social support [18].

### 2.4. Statistical Analysis

In this study, a two-tailed significance level of overall *p* < 0.05 was considered statistically significant. SAS, version 9.4 (SAS Institute Inc.), was used. Continuous data are shown as the means ± standard deviation. Two-sample Wilcoxon tests for two groups were applied to evaluate different across groups according to various variables, such as sex, living in rural areas, educational level, marital status, medical insurance, monthly income, substance dependence (smoke, alcohol drink), hypertension, diabetes, atrial fibrillation, infarct location, family function, and social support and subscales of SCL-90-R. Subgroup analyses were performed for young adult stroke patients with and without psychological symptoms. We performed multivariable logistic regression analyses using stepwise variable selection, and all variables were entered into the model to explore independent impact factors for psychological status. *p* < 0.15 was used for variable selection.

## 3. Results

### 3.1. Comparisons between Young Ischemic Stroke Patients and Age-Matched Young Healthy Controls

In this sample, a total of 364 young adult stroke patients were included, with an age of 31.8 ± 6.3 years (from 20 to 44 years). The positive detection rate of psychological abnormalities in young stroke patients was 22.3% (81/364 cases), with the reference of 160 as the cut-off value in China [28]. The SCL-90-R total score and subfactors were presented in Table 1. In comparison with the age-matched healthy controls during the same study period, the young patients in our study had higher scores on psychological variables, including somatization, obsessive-compulsive, interpersonal sensitivity, depression, anxiety, hostility, phobic anxiety, paranoid ideation, and psychoticism (*p* < 0.01 or 0.05).

### 3.2. Clinical Characteristics between Young Ischemic Stroke Patients with and without Psychological Symptoms

Based on the SCL-90-R total score of 160 as a cut-off, all patients were classified into two subgroups as patients with and without psychological symptoms showing in Table 2. Marital status (*p* = 0.03), hypertension (*p* = 0.01), infarct size (*p* = 0.01), and percentage of patients with different levels of FFAS scores (*p* < 0.01) were found significantly different between two subgroups.

### 3.3. Multivariate Regression Analysis

The multivariate logistic regression analyses (Table 3**)** showed that the family dysfunction (odds ratio [OR], 2.50, 95% confidence interval [CI], 1.71 to 3.54; *p* < 0.01), having hypertension (OR, 3.27; 95% CI, 1.92 to 4.27; *p* = 0.02), and ≥20mm^3^ infarct size (OR, 2.39, 95% CI: 1.53 to 3.45, *p* < 0.01) were risk factors for psychological symptoms among young ischemic patients.

In depression models, being single (OR, 1.23, 95% CI: 1.03 to 1.54, *p* = 0.01), the family dysfunction (OR,1.21, 95% CI: 1.05 to 1.45, *p* = 0.03), and ≥20 mm^3^ infarct size (OR, 1.74, 95% CI: 1.14 to 3.13, *p* = 0.02) were selected as independent factors for patients with psychological symptoms. For somatization and anxiety, the family dysfunction (OR, 2.32, 95% CI: 1.51 to 2.80, *p* < 0.01) and hypertension (OR, 2.41, 95% CI: 1.54 to 3.46, *p* = 0.03) were predictors among patients with psychological symptoms, respectively.

## 4. Discussion

The study showed that young ischemic adult stroke patients at three-month timepoint after their stroke had obvious psychological symptoms with an incidence of 22.3%, and the patients with psychological symptoms had higher percentages of married status, hypertension, family dysfunction, and large infarct size. The family dysfunction, having hypertension, and larger infarct size were prominently risk factors for those young patients developing psychological symptoms at three months after stroke.

Around one-fifth of patients with young ischemic stroke had psychological symptoms after three months of onset. This means that those young stroke patients are commonly comorbid with psychological abnormalities, which may negatively affect their quality of life and recovery outcome [5, 32] and might develop into various mental disorders after stroke [1]. Unlike older adults, as a particular social group, young people bear greater social responsibility. Therefore, it is of great significance to formulate strategies for youth stroke health care, which needs physical rehabilitation and psychological support. This concept of mixture intervention and rehabilitation needs to be gradually established for young stroke patients.

Our study found that young adult stroke patients with psychological symptoms had larger infarct size and higher percentages of having hypertension and family dysfunction than those in patients without psychological symptoms. There are no differences on clinical features, including infarct locations, NIHSS score, mRS score, BI score, diabetes, atrial fibrillation, smoking, and drinking, and social supports, including subjective support, objective support, and utilization of support. These results indicated that two groups with and without psychological symptoms had similar disease features when their acute stages of stroke and the same social supports around them after three months. We further revealed that large infarct size, hypertension, and family dysfunction at the onset of stroke were risk factors for having psychological abnormalities among patients. Being single, the family dysfunction, and large infarct size were risk predictors for patients with psychological symptoms to have depressive symptoms. And the family dysfunction was a risk of emerging somatization and hypertension for anxiety in patients with psychological symptoms. These findings implied that the aforementioned variables might be associated with future intervention targets for young stroke patients.

Our results were consistent with the previous reports that a good family function is a crucial protector for family members to cope with emergencies and alleviate their psychological stressors [33, 34]. Importantly, the family function is closely related to individual health status, disease occurrence, and recovery [34]. The possible reasons for family function's role in an individual psychological situation may involve that family members have close relationships with each other and have subjective satisfaction with family functions. The close relations among family members do benefit to reduce the psychological stress and avoid the occurrence of negative emotions. Furthermore, the patient in good family function can obtain other family members' immediate assistance and relieve his/her psychological stress associated with stroke.

Our study did not find that social support was different among two groups in young adult stroke patients. This may indicate that subjects in our study have necessary social support for their daily life. Indeed, satisfactory social support means that individuals could obtain social support from the outside when they need help [35] and avoid the occurrence of adverse psychological problems [36, 37]. In addition, social support theory holds that social support can alleviate individual stress in adverse events and is a protective factor for individuals' physical and mental development [36–38]. Moreover, social support is closely related to the individual's ability to respond to adverse events [39].

The study had some limitations. First, the study was a cross-sectional design, which is hard to verify the causal relationships of hypertension, infarct size, family functioning, and psychological status in young stroke patients. Second, abnormal psychological status may cause poor family function. Therefore, longitudinal studies are needed to clarify the causality in young stroke patients. Third, the study had an uneven number of samples in subgroups divided by clinical variables, especially marital status. Therefore, the results of the spousal situation in this study will need to be further verified. These limitations need to be further explained for developing effective strategies for young stroke patients.

The study provided meaningful evidence for young stroke patients for their further intervention, and some strengths should be emphasized. Our study is the first report on young Chinese stroke patients who had abnormal psychological status at three months after their stroke. The results benefit these patients' recovery after stroke via caring for psychological status. In addition, our study was conducted in outpatient clinic settings. The results had general application into other common outpatient settings.

## 5. Conclusions

In conclusion, young Chinese adult stroke patients had obvious psychological symptoms at three-month timepoint after their stroke, severe family dysfunction, hypertension, and large infarct size were risk predictors of emerging psychological abnormalities in Chinese young adult stroke patients three months later after their stroke. Therefore, further prevention and intervention strategies on psychological symptoms should focus on bettering family function, controlling hypertension, and positively intervening in primary vascular diseases associated with young ischemic stroke, to enhance their recovery after stroke.

## Figures and Tables

**Table 1:** Comparisons of SCL-90-R between young ischemic stroke patients and age-matched young healthy controls.

Features	Healthy (*n* = 384)	Patients (*n* = 364)	*p* ^1^
Age (years), mean ± SD	31.9 ± 6.1	31.8 ± 6.3	0.85
Male sex, % (*n*)	33.8 (130)	36.5 (133)	0.44
Urban residents, % (*n*)	92.4 (355)	97.2 (354)	0.52
Senior high school or higher, % (*n*)	93.5 (359)	93.1 (339)	0.84
Married, % (*n*)	42.2 (162)	70.3 (256)	<0.01
Had medical insurance, % (*n*)	98.7 (379)	98.6 (359)	1.00
Monthly income >6000 yuan, % (*n*)	57.3 (220)	56.9 (207)	0.91
Total SCL-90-R scores, mean ± SD	98.6 ± 16.9	147.4 ± 26.1	<0.01
Subscales of SCL-90-R			
Somatization, mean ± SD	1.1 ± 0.4	1.8 ± 0.5	<0.01
Obsessive-compulsive, mean ± SD	1.2 ± 0.3	1.7 ± 0.3	<0.01
Interpersonal sensitivity, mean ± SD	1.2 ± 0.3	1.5 ± 0.2	<0.01
Depression, mean ± SD	1.1 ± 0.3	1.7 ± 0.3	<0.01
Anxiety, mean ± SD	1.1 ± 0.3	1.8 ± 0.5	<0.01
Hostility, mean ± SD	1.0 ± 0.3	1.8 ± 0.4	<0.01
Phobic anxiety, mean ± SD	1.0 ± 0.4	1.8 ± 0.4	<0.01
Paranoid ideation, mean ± SD	1.0 ± 0.4	1.1 ± 0.1	0.02
Psychoticism, mean ± SD	0.9 ± 0.2	1.4 ± 0.1	<0.01

Abbreviations: SCL-90-R: Symptom Checklist 90 Revised; SD: standard deviance; ^1^*p* value was obtained using chi-square tests or Fisher's exact tests for categorical variables and Mann–Whitney *U* tests for continuous variables.

**Table 2:** Comparisons on clinical characteristics between young ischemic stroke patients with and without psychological symptoms.

Characteristics	Patients without psychological symptoms (*n* = 283)	Patients with psychological symptoms (*n* = 81)	*p* ^1^
Age (years), mean ± SD	31.8 ± 6.3	31.9 ± 6.2	0.46
Male sex, % (*n*)	37.1 (105)	34.6 (28)	0.68
Urban residents, % (*n*)	97.2 (275)	97.5 (79)	1.00
Senior high school or higher, % (*n*)	93.6 (265)	91.4 (74)	0.47
Married, % (*n*)	67.5 (191)	80.2 (65)	0.03
Had medical insurance, % (*n*)	98.9 (280)	97.5 (79)	0.34
Monthly income>6000 yuan, % (*n*)	55.8 (158)	60.5 (49)	0.45
Smoker, % (*n*)	23.3 (66)	14.8 (12)	0.10
Drinker, % (*n*)	24.4 (69)	29.6 (24)	0.34
Hypertension, % (*n*)	10.2 (29)	21.0 (17)	0.01
Diabetes, % (*n*)	12.4 (35)	12.4 (10)	1.00
Atrial fibrillation, % (*n*)	20.1 (57)	18.5 (15)	0.75
Infact location, % (*n*)			0.06
Cortex	32.5 (92)	21.0 (17)	
White matter lesions	4.6 (13)	0.0 (0)	
Basal ganglia + thalamus	32.5 (92)	39.5 (32)	
Brain stem	23.3 (66)	29.6 (24)	
Cerebellum	7.1 (20)	9.9 (8)	
Infarct size mm^3^, mean ± SD	20.63 ± 30.48	31.87 ± 43.71	0.01
NHISS score, mean ± SD	2.8 ± 3.3	2.6 ± 3.2	0.61
mRS score, mean ± SD	2.5 ± 0.8	2.5 ± 0.7	0.78
Bl score, mean ± SD	82.9 ± 24	81.7 ± 27.6	0.70
Total SCL-90, mean ± SD	134.8 ± 7.6	191.6 ± 18.5	<0.01
FFAS total score, mean ± SD	4.5 ± 1.5	4.4 ± 2.2	0.75
7-10	15.6 (44)	24.7 (20)	<0.01
4-6	52.3 (148)	30.7 (25)	
0-3	32.2 (91)	44.4 (36)	
SSRS total score, mean ± SD	34.7 ± 10.2	33.2 ± 11.3	0.27
<20	9.2 (26)	7.4 (6)	0.09
20-30	22.6 (64)	34.6 (28)	
>30	68.2 (193)	28.0 (47)	
Subjective support, mean ± SD	20.1 ± 5.2	19.3 ± 5.8	0.22
Objective support, mean ± SD	8.1 ± 3.3	7.5 ± 3.6	0.16
Utilization of support, mean ± SD	6.5 ± 2.0	6.4 ± 2.3	0.85

Abbreviations: SD: standard deviance; NIHSS: National Institute of Health Stroke Scale; mRS: the modified Rankin Scale; BI: Barthel Index; FFAS: the Family function assessment scale; SSRS: the Social support rating scale; ^1^*p* was obtained using chi-square tests or Fisher's exact tests for categorical variables and Mann–Whitney *U* tests for continuous variables.

**Table 3:** Outcomes of psychological manifestations via multivariate logistic regression analyses using stepwise variable selection.

Variables	OR (95% CI)	*p*
Model for SCL-90-R		
Family function (moderate and serious dysfunction vs. good)	2.50 (1.71, 3.54)	<0.01
Hypertension (yes vs. no)	3.27 (1.92, 4.27)	0.02
Infarct size (≥20 vs. <20 cm^3^)	2.39 (1.53, 3.45)	<0.01
Model for depression		
Marital status (single vs. married)	1.23 (1.03, 1.54)	0.01
Family function (moderate and serious dysfunction vs. good)	1.21 (1.05, 1.45)	0.03
Infarct size (≥20 vs. <20 cm^3^)	1.74 (1.14, 3.13)	0.02
Model for somatization		
Family function (moderate and serious dysfunction vs. good)	2.32 (1.51, 2.80)	<0.01
Model for anxiety		
Hypertension (yes vs. no)	2.41 (1.54, 3.46)	0.03

Abbreviations: OR: odds ratio; CI: confidence interval; SCL-90-R: Symptom Checklist 90 Revised.

## Data Availability

The materials in this manuscript are available from the corresponding author on reasonable request.
